This article has been retracted.

# Design of Faster R-CNN-Based Fault Detection Method for Subway Vehicles

**DOI:** 10.1155/2022/1400658

**Published:** 2022-07-08

**Authors:** Hanlin Ma, Mingyang Yao

**Affiliations:** ^1^School of Power Technology, Liuzhou Railway Vocational Technical College, Liuzhou Guangxi 545616, China; ^2^School of Automatic Control, Liuzhou Railway Vocational Technical College, Liuzhou Guangxi 545616, China

## Abstract

A substantial amount of maintenance and fault data is not properly utilized in the daily maintenance of pantographs in urban metro cars. Pantograph fault analysis can begin with three factors: the external environment, internal flaws, and joint behavior. Based on the analysis of pantograph fault types, corresponding measures are proposed in terms of pantograph fault handling and maintenance strategies, in order to provide safety guarantee for the safe and effective realization of rail transit vehicle speed-up and also provide reference for the maintenance and overhaul of pantographs. For the problem of planned maintenance no longer meeting current pantograph maintenance requirements, a defect diagnosis system based on a combination of faster R-CNN neural networks is presented. The pantograph image features are extracted by introducing an alternative to the original feature extraction module that can extract deep-level image features and achieve feature reuse, and the data transformation operations such as image rotation and enhancement are used to expand the sample set in the experiment to enhance the detection effect. The simulation results demonstrate that the diagnosis procedure is quick and accurate.

## 1. Introduction

The development of society and urbanization construction continues to deepen and improve people's material living standards, so that they improve the requirements for quality of life. In addition, the progress of society has led to the development of China's transportation industry, such as the development of China's metro rail transportation field is in a better situation, and the station has a high flow of people. In this development context, to create a safe travel environment for the public, for metro transportation operations, it is necessary to focus on the operation, monitoring, and maintenance management of station equipment, timely understanding of equipment safety conditions, the discovery of faults, and effective handling of problems, to ensure the safe operation of metro transportation [1–3]. With the continuous progress of rail transportation technology in China, the development of rail transportation operating vehicles from steam locomotives to internal combustion locomotives and electric locomotive traction is particularly notable. Electrified railroads occupy a large part of China's rail traffic mileage, for the routine and troubleshooting of rail vehicles which are particularly important. In the existing electrified railroad operation lines, according to the statistics of various accidents in the past years, the vehicle equipment failures caused by pantographs account for a relatively large proportion. Pantograph is an important part of the vehicle but also is in direct contact with the contact network part, in the vehicle high-speed travel by wear and tear, and has a high probability of failure [4–6]. Rail vehicle power supply and operation disruptions have a significant impact on line transportation order and are a major issue for rail cars. As a result, understanding and treating common pantograph failure is critical for the safe and reliable operation of rail transit. The subway fault diagnosis system is shown in Figure 1.

China's environmental monitoring equipment industry started late, environmental monitoring equipment is mostly produced by small and medium-sized enterprises, and products are basically concentrated in the low-grade environmental monitoring equipment, still far from being able to meet the needs of the development of China's environmental monitoring work, mainly in terms of poor product quality, short service life, unstable performance, and high failure, which leads to low frequency of environmental monitoring, sampling errors, and inaccurate monitoring data can not. This leads to low frequency of environmental monitoring, large sampling errors, and inaccurate monitoring data and cannot reflect the environmental quality in a timely manner. Therefore, it is of great significance to strengthen the equipment fault monitoring to ensure the normal operation of the equipment and improve the safety and reliability of the equipment [7, 8]. Currently, equipment defect detection research is mostly focused on the analysis of infrared thermal pictures of equipment. The maximum temperature value around the equipment is calculated in the detection of thermal faults in power equipment by identifying the power equipment in the thermal image based on the shape characteristics of the equipment, the diagnosis is made after correcting for various influencing factors, and satisfactory results are achieved. It is also possible to achieve high detection accuracy and robustness in the detection of thermal faults in power equipment by comparing the results obtained from the temperature information in the alignment area of the infrared image with each other. Due to the influence of environmental temperature and other factors on infrared thermal images, these methods still have great limitations. With the wide application of deep learning in the field of target detection, faster R-CNN algorithm, as one of the classical algorithms in this field, has high recognition accuracy and fast detection speed and has been widely used in vehicle detection, static aircraft detection, commodity image detection, etc. [9].

In this paper, we propose a faster R-CNN-based fault detection and recognition method for environmental monitoring equipment, which applies faster R-CNN to the fault detection of environmental monitoring equipment. Then, through the equipment fault online detection system, we can realize online real-time monitoring, so that we can get the information whether the equipment has a fault in time and effectively and notify the relevant staff [10, 11]. This paper mainly verifies the feasibility of deep learning in environmental monitoring equipment fault identification from three aspects: equipment switches status identification, equipment indicator abnormality identification, and equipment display abnormal data identification, which effectively solves the problem of fault detection of environmental monitoring equipment, saves human and material resources, and further realizes the automatic detection of equipment. For the problem of low detection accuracy in the case of small contact network pantograph fault image samples, a dense convolutional neural network model is introduced as the feature extraction network of the faster R-CNN model for pantograph fault detection. The fused multilevel target features are extracted to improve the recognition capability of the model, and the sample set is expanded by using data transformations such as image rotation and enhancement to further improve the detection performance of the model. Through the experimental detection of the collected contact network pantograph images, the faster R-CNN model with a backbone network achieves good detection results in terms of both detection accuracy and speed.

The following is the paper's organization paragraph: Section 2 discusses the overall research related work. The method of the proposed concepts of this paper is examined in Section 3. The calculation example is discussed in Section 4. Finally, the research job is completed in Section 5.

## 2. Related Work

### 2.1. Intelligent Detection of Subway Faults

Research on fault detection and intelligent diagnosis system of metro electromechanical equipment and monitoring function are as follows: dynamic image display function. Dynamic image display function, the fault detection and intelligent diagnosis of subway electromechanical equipment work, can fully display the operation of the equipment [12–14]. During the actual work of the staff, use the system operation to analyze the data information of the equipment work as well as the operation safety, use the mouse to link to the property bar of the equipment, find the operation work information of the equipment, and set the corresponding authority. Alarm function is as follows: when problems occur during the operation of electromechanical equipment in the system, the intelligent diagnosis system can give priority to the alarm processing of faults, display the faults visually and comprehensively in the human-machine interface, and take effective measures to solve the actual problems by combining the severity of the problems. Control function is as follows: the control function of electromechanical equipment. Through the intelligent diagnosis system, the fault personnel can directly log into the metro station control system and use the system's assigned authority to effectively control the electromechanical equipment. The functions of electromechanical equipment are group control function, control function of single machine equipment, and enthalpy control function. Mode of control [15, 16]: combined with the actual application of electromechanical equipment in demand, the staff selects the appropriate mode to set each parameter of the system, selects the appropriate parameters, and controls in this mode. For example, in the case of BAS modal control, the staff can optimize the parameters according to their own needs and set the correct parameter values, which can ensure the optimal operation of different modes. Display function: metro electromechanical devices and equipment, in the fault detection phase, the system can be displayed in the interface using human-computer interaction technology [17]. This enables staff to grasp the dynamic operation effect and parameters of each device, use the interface to present operating data, judge the device's performance in a timely manner, identify safety threats, offer relevant control instructions in a timely manner, and apply effective methods to solve.

The subway fault handling process is shown in Figure 2. There is the fault detection logical architecture scheme of the subway electromechanical equipment, fault monitoring and intelligent diagnosis system, manipulation, and maintenance of electromechanical devices through intelligent means, and the entire system framework covers data acquisition system, diagnosis system, transmission system, decision-making system, and various parts of the application layer. The abovementioned parts are also the main elements of the system logical architecture, and attention should be paid to the need to cover during the design of the program. Data acquisition system designs program data acquisition layer, detecting the main sections of the equipment using the actual operational condition of electromechanical equipment and the acquisition of fault information, rather than equipment running speed, temperature, and vibration, etc. At the same time, for each intelligent equipment, screen doors, subway elevators, and other equipment, intelligent detection objectives can be achieved, through the interface of data, can directly obtain the detection data, through the sensing equipment to control the temperature during the operation of the equipment and vibration information, and can ensure the real-time information collection [18]. The data analysis system is designed to obtain data and information during the operation of the system, to analyze it in-depth, to build algorithms for data analysis and a database of fault information, to facilitate the accurate acquisition of fault characteristics and signals, and to analyze the causes of faults and future development directions. The data analysis system can also effectively analyze the spectrum of equipment vibration time, accurately determine the existing problems, and complete the intelligent diagnosis and processing of electromechanical devices. The data transmission system uses network technology to achieve equipment diagnosis and fault analysis, the field data transmission to the subway station, and maintenance management office, facilitating the timely transmission of effective information to the staff, as equipment and system operation, the implementation of management work. At the same time, standardized and open network protocols are set for data transmission to facilitate timely access to data information by staff [19–21].

### 2.2. Subway Fault Intelligent Diagnosis

The function of the decision evaluation system is to store the expert system for the maintenance of metro devices, to accurately evaluate the state of the equipment, historical data, and maintenance information, to make a comprehensive judgment on the operation of the equipment, to assess the future development situation, to reduce the difficulty of the maintenance work for the staff, and to do early warning work. At the same time, it is also able to combine the actual operation of the set, optimize the plan of maintenance, and strengthen the maintenance efficiency of electromechanical equipment. Application system functions as follows: providing a large amount of maintenance information and technical support, providing effective information for electromechanical equipment maintenance work, using the interface of human-computer interaction, and showing equipment operation data and information. The data and information of equipment operation, various resources, and maintenance data are recorded, accurately counted, queried, stored, and processed in a timely manner. In addition, it can also provide data information printing services for practical applications based on specific work requirements [22].

The structure design of fault detection and intelligent diagnosis system of metro electromechanical equipment is divided into a three-level detection and two-level management structural framework based on the above logical system design and combined with the specific functional requirements of the system. The main content covers the line maintenance center system, the maintenance of the working area of the accumulation equipment, and the three-level detection of the equipment. The hierarchical management and data transmission of the system can be realized by using network information technology and software platform, and through the framework mode of hierarchical distribution, this structure is more flexible in deployment and easy to expand. In addition, the application of Web technology reduces the difficulty of staff work, timely access to fault detection, and intelligent diagnosis of data information. Line maintenance of the central system, set in the subway line vehicle section of the maintenance center location, the use of network data transmission and information management methods, intelligent processing of data information in operation, combined with data implementation equipment management, and detection of information in the whole line, can determine the fault for the future development trend, to achieve the alarm function of the fault, to create favorable conditions for the work of the staff, accurate find the cause and location of the fault, the location, fault characteristics, and other information, transported to the system's database center, and can achieve the goal of information-based maintenance of equipment. The electrical and mechanical work area system combines the actual operation needs of the subway, and based on past experience, the system treats four to six stations as intervals and installs electrical work areas at each interval point to facilitate maintenance and management in conjunction with the actual situation and to determine the factors that produce faulty equipment. In addition, the fault personnel is able to operate the faulty equipment and obtain the operation information and data of the accumulated equipment inside the work area and associate it with the printer to realize the printing and maintenance of information [23].

## 3. Methods

### 3.1. Analysis of Faults

There are many different types of pantograph structures, which can be classified as pop-up and inflatable based on their transmission methods, single-arm and double-arm based on their arm shapes, high-speed and normal-speed based on their usage speeds, and single pantograph and double pantograph based on the number of pantograph frames. Single-arm pantographs are currently the most common on China's rail vehicles. Pantograph is mainly composed of bow head, frame, chassis, and driving mechanism. The chassis support frame is installed in the upper part of the vehicle through the insulator, and the support frame supports the pantograph head by lifting the bow spring. From the structural point of view, the whole frame is composed of 2 four-bar mechanisms, and the drive mechanism is installed in the lower arm of the frame to realize the up-and-down movement of the pantograph. When the pantograph head is in operation, the height of the contact network varies, and the head's basic level must be maintained as the pantograph moves. If the pantograph head cannot maintain horizontal movement, the contact surface between the contact wire and the slide plate cannot be continuous, which may cause the pantograph head to wear out and lead to the contact wire going offline.  Figure 3 shows the structure of single arm pantograph.

Here are the following parts of the pantograph: (1) carbon slide plate, (2) bracket, (3) balance bar, (4) upper frame, (5) hinge seat, (6) lower arm bar, (7) sector plate, (8) buffer valve, (9) drive cylinder, (10) piston, (11) lowering bow spring, (12) link insulator, (13) slip ring, (14) link rod, (15) support insulator, (16) raising bow spring, (17) bottom frame, and (18) push rod. After the pantograph of a subway rail vehicle is raised and meets the overhead contact network, current is obtained from the contact network and transmitted to the vehicle electrical system. The current flows from the contact network to the head of the bow and flows into the bottom frame through the upper arm bar and lower arm bar in turn and finally enters the vehicle electrical system through the connecting plate and roof bus. When raising the bow, start the air compressor, when the rated working air pressure of the pantograph is reached, press the button to raise the bow, the compressed air enters the air spring from the solenoid valve and control box, the pneumatic equipment pushes the wire rope to drive the movement of the lower arm bar and holds up the upper arm bar of the pantograph, and the bow head moves smoothly to the height of the contact network to complete the raising of the bow. When lowering the bow, the pantograph falls smoothly to the rubber stop on the bottom frame with the help of gravity, and the hydraulic damper after the pantograph control box releases the compressed air in the air spring. According to the summary analysis of the daily maintenance records of this type of pantograph, combined with the failure mode of single-arm pneumatic pantograph and its mechanism analysis, the failure forms of pantograph can be summarized into five types of pantographs: pantograph cannot be raised, status display mismatch, bow network arc pulling, pantograph parts damage, and pantograph cannot respond.

### 3.2. Model Structure

The faster R-CNN model consists of two modules: the candidate region proposal network (RPN) and the fast R-CNN detection module. It can be subdivided into four parts: the first part is the convolutional neural network, which is mainly used to extract the features of the input pantograph images, the VGG16 network is used, and the feature map is the extracted pantograph image features; the second part is the region proposal network (RPN), which is mainly used to generate the candidate regions and initially. The third part is the region of interest pooling (RoI pooling), which is used to convert the input candidate regions of different sizes into fixed sizes and output them as vectors of the same length; the fourth part is the classification and border regression, which is used to output the pantograph state classes to which the candidate regions belong and the exact positions of the candidate regions in the original The fourth part is classification and border regression, which is used to output the pantograph state category to which the candidate region belongs and the exact position of the candidate region in the original image. The proposed model architecture is shown in Figure 4.

### 3.3. Pretrained Convolutional Neural Network Models

Pretrained models are models created by previous authors to solve similar problems. Using pretrained models can save a lot of time by not having to train a new model from scratch. Varied convolutional neural network models, on the other hand, can have different effects on detection speed, accuracy, and other factors. The authors of the original faster R-CNN paper extract picture features using the Ziller and Fergus network model and the visual geometry group network model as the backbone network of faster R-CNN. Among them, ZFNet mainly adjusts the parameters of AlexNet by reducing the convolutional kernel and step size so that the network can extract more detailed features and thus improve the performance of the network; while in VGGNet, the convolutional layers all use the same convolutional parameters, the pooling layers all use the same pooling parameters, and its network consists of several 3 × 3 convolutional layers and 2 × 2 pooling layers stacked repeatedly. The network structure is simple, but uses more parameters, has a higher memory occupation, and requires more computational resources.

### 3.4. RPN Network

In training the RPN network, the above pretrained network model is directly used to initialize the RPN, and the pantograph feature maps extracted by the pretrained network model are input to the RPN network. The RPN network generates region proposals on the feature maps using sliding windows of different sizes and dimensions, and then the region proposals are input to the classification layer and the regression layer, respectively. In the classification layer, a normalization function (Softmax) is used for target detection to determine whether the proposed region contains a pantograph target, while the regression layer is used to calculate the offset of the proposed region bounding box regression, which is used to adjust the anchor points to obtain an accurate target candidate region. The RPN network uses a multitask loss function to calculate the loss, including classification loss and border regression loss, and the formula is defined as

(1) $$\begin{array}{c} \begin{array}{c} L\left(\left\{P_{i}\right\},\left\{t_{i}\right\}\right)=\frac{1}{N_{\text{cls}}}\underset{i}{\sum }\;L_{\text{els}}\left(P_{i},P_{i}^{*}\right)+\lambda \frac{1}{N_{\text{reg}}}\\ \underset{i}{\sum }\;P_{i}^{*}L_{\text{reg}}\left(t_{i},t_{i}^{*}\right), \end{array}, \end{array}$$

where *i* is the index of anchors in small batch training, *P*_*i*_ denotes the probability that an anchor is a target, *P*_*i*_^∗^ denotes the presence or absence of a target for the anchor (1 for the presence of a target, 0 for the absence), *t*_*i*_ denotes the 4 parameterized coordinate vector of the predicted bounding box, *t*_*i*_^∗^ denotes the coordinate vector of the labeled bounding box, *N*_cls_ denotes the batch size (generally taken as 256), *N*_reg_ denotes the number of anchors, *λ* is the balance parameter and is set to 10 by default; the outputs of classification and regression layers consist of {*P*_*i*_}, {*t*_*i*_}, respectively, Lcls is the classification loss, which denotes the logarithmic loss of two classes (target and nontarget), and Lreg is the regression loss, defined as

(2) $$\begin{array}{c} \begin{array}{c} L_{\text{reg}}\left(t_{i},t_{i}^{*}\right)=\\ R\left(t_{i}-t_{i}^{*}\right)=\left\{\begin{array}{cc} 0.5{\left(t_{i}-t_{i}^{*}\right)}^{2} & \text{ if }\left|x\right|<1.\\ \left|t_{i}-t_{i}^{*}\right|-0.5 & \text{ otherwise } \end{array}\right. \end{array} \end{array}$$

### 3.5. Fast R-CNN

The fast R-CNN module consists of two parts: RoI pooling and classification regression; in faster R-CNN, the input of fast R-CNN module is the candidate regions output by RPN network. Features protect the complete structure and original shape information of the input image. Each feature vector is then fed into multiple fully connected layers behind and finally output by two subconnected layers of the same level, the classification layer and the regression layer, similar to the output of RPN networks, except that the output of the classification layer is the probability value of the candidate region belonging to each category, and the output. The loss function used in the fast recurrent-convolutional neural network (R-CNN) module is similar to that of the RPN module, except that the binary classification is changed to multiclassification, and only the regression loss of the candidate regions predicted to be labeled classes is considered. The DenseNet model borrows the idea of the RPN model, which also connects the features of the front layer of the network to the back layer, but unlike ResNet, it adopts a new network structure, in which the core idea of the ResNet model is to establish a “short-circuit connection” between the front layer and the back layer, using the connection method of element-level summation, whereas DenseNet establishes a dense connection between all the preceding layers and the following layers, in which the input of each layer of the network is the concatenation of the output of all the preceding layers within a module. This difference can also be visualized from the transfer functions of the two network structures: The transfer function of the ResNet network is

(3) $$\begin{array}{c} x_{l}=H_{l}\left(x_{l-1}\right)+x_{l-1}. \end{array}$$

The transfer function of the DenseNet network is

(4) $$\begin{array}{c} x_{l}=H_{l}\left(\left[x_{0},x_{1},\cdots ,x_{l-1}\right]\right). \end{array}$$

The dense connection has many advantages, it can directly parallelize the features from different layers to achieve feature reuse, which is more conducive to information transfer, and it can mitigate the gradient disappearance during back propagation and reduce the problem of easy overfitting due to the small sample size of the network training. The schematic diagram of the densely connected network is shown in Figure 5.

### 3.6. Data Preprocessing

Since the collected pantograph initial state data involve many parameter variables, this paper selects the principal element analysis method to reduce its dimensionality. The principal element analysis (PCA) method is a transformation method that reflects multiple relevant variables with relatively few feature variables but carrying enough information. On the premise of ensuring the correct diagnosis rate, redundancy and noise are eliminated, and then the dimensionality reduction of the original feature data variables is realized to reduce the diagnosis time consuming and improve the diagnosis efficiency. The calculation process is as follows:

1. Construct the original variable matrix *X*_0_ ∈ *R*. the rows *x*_*i*_ of the matrix correspond to the original data samples, and the columns *x*_*j*_ of the matrix correspond to the different measured. Since the different magnitudes of the initial data can lead to serious dispersion of the variable results, the observation samples need to be standardized
2. The covariance solution of the processed matrix *X*_0_ is performed, i.e., the calculation of the correlation coefficient matrix *R*; that is,

(5) $$\begin{array}{c} r_{jk}=\frac{\sum_{k=1}^{n}\;\left(x_{ki}-x_{i}\right)\left(x_{ki}-x_{j}\right)}{\sqrt{\sum_{k=1}^{n}\;\left(x_{ki}-x_{i}\right)\sum_{k=1}^{n}\;{\left(x_{ki}-x_{j}\right)}^{2}}}. \end{array}$$

(3) Solve the covariance matrix to obtain the eigenvalue eigenvectors. Calculate the value of the eigenequation |*λI* − *R*| = 0 and order the eigenvalues sought, from largest to smallest, noted as *λ*1 ≥ *λ*2 ≥ , ⋯, ≥*λm* ≥ 0, corresponding to the eigenvectors *I*_1_, *I*_2_, *…*, *I*_*m*_
(4) The feature vectors are transformed into principal elements, and the contribution rate and cumulative contribution rate of the principal elements are calculated:

(6) $$\begin{array}{c} T_{j}=I_{1}X_{1}+I_{2}X_{2}+\cdots +I_{m}X_{m}, \end{array}$$

where *T*_*j*_ is the *j*-th principal element, representing the projection of matrix *X* on the corresponding principal element feature vector, and the larger the corresponding coverage, the longer its projection length will be. If the principal element *T*_*j*_ decreases, then *I*_1_ is the direction that covers the widest degree of information.

(5) Calculate the cumulative contribution rate *α*

(7) $$\begin{array}{c} \begin{array}{c} T_{j}=\frac{\lambda_{j}}{\sum_{j=1}^{p}\;\lambda_{j}}\times 100\%,\\ \alpha =\frac{\sum_{s=1}^{i}\;\lambda_{s}}{\sum_{j=1}^{p}\;\lambda_{k}}\times 100\%. \end{array} \end{array}$$

## 4. Experiments and Results

### 4.1. Data Set

The pantograph image data for this experiment mainly came from the pantograph images collected by the contact network suspension state detection and monitoring device (4C device), and the samples were divided into three categories by analyzing the pantograph morphology in the images: the first category was normal pantographs, the second category was bent pantographs, and the third category was broken pantographs. 3. 2 Data set processing. This experiment got a total of 3563 contact network photos taken by the 4C device. After choosing and eliminating the blurred and pantograph-free samples from the 3563 contact network images received from 4C equipment, 1672 good samples were obtained. The database details are shown in Table 1. To increase the diversity of samples and improve the accuracy of pantograph identification and fault detection, this paper expands the sample set by rotating the original images clockwise by 30°, 60°, and 90°, enhancing the brightness to 1.2 times, attenuating it to 0.8 times, and adding pepper noise with a density of 0.01 and other six data transformation operations. A total of 1672 × 7 = 11704 samples of the data set were obtained after processing. Considering that the actual detection process does not require too high a resolution, and that the pretrained models used in this paper were all trained on the PASCALVOC dataset; the resolution of the image aspect was scaled by 10 times each for the compression process, and the compressed image aspect was between 300 and 600 pixels. Then, all samples in the dataset were labeled using the LabelImg standard tool. The category labels of normal pantograph, bending deformation pantograph, and broken pantograph are labeled as “zcdx,” “xbdx,” and “dkdx,” respectively. Then, the samples of the data set were randomly divided into training and test sets in the ratio of 7 : 3, where data set 1 is the original data sample; data set 2 is the data sample after adding the data transformation process.

### 4.2. Experimental Setup

This experiment is conducted under Windows 10 Home Edition operating system, based on Intel(R) Core (TM) i5-8300H CPU2, 3GHz (8GByte running memory), and NVIDIAGeForceGTX1050TiGPU (4GByte running video memory) hardware device to build Google TensorFlow graph (TensorFlow) deep learning framework, using the Python programming language, using the faster R-CNN architecture to implement the training of network models, using the divided dataset as training samples, and using VGG16, ResNet101, and DenseNet121 as the backbone network of the faster R-CNN in turn to train the pretrained. The training of the contact network pantograph identification and fault detection network model is accomplished using the faster R-CNN model. In this paper, the end-to-end training method is used to share convolutional features, and the stochastic gradient descent (SGD) algorithm is used to optimize the model, with the maximum number of iterations set to 40,000, the initial learning rate set to 0.001, the momentum factor set to 0.9, and the learning rate adjusted to 0.0001 when the number of iterations reaches 20,000.0001; meanwhile, output its average loss every 1000 times and stop training when the loss function converges, and the number of iterations reaches 40,000, using VGG16, ResNet101, and DenseNet121 as the backbone network to train the faster R-CNN model. After training, the trained model parameters are saved, and the model effect is further validated using the divided test set, preserving the four sample target classes with confidence levels larger than 0.5.  Figure 6 depicts the loss degradation during training, while Figure 7 depicts the improvement in performance.

### 4.3. Experimental Results

The metrics for measuring the goodness of the model in this research are average precision (AP) and mean accuracy (mAP), where AP is calculated based on the precision rate *P* and recall rate *R*, if the classification results are represented as in Table 2.

In this paper, the same computer is used for training and testing of all samples. In order to improve the accuracy of model recognition, multiple data transformations are used to expand the sample set, and different network models are used as the backbone network of the faster R-CNN model, while mAP is cited to visually compare the recognition accuracy of each network model, combined with the recognition speed, to select the best applicable contact network pantograph fault detection. The network models are selected as the best network models for pantograph fault detection.4. 1 Comparison of recognition results of three network models. The faster R-CNN models with VGG16, ResNet101, and DenseNet121 as the backbone networks are trained using the training set of the original dataset1 in turn, and the training methods in Section 3.3 are used for all training methods. The resulting models were then evaluated against the test set of datasets 1, and the A*P* values of each category were produced based on each model's detection outcomes and combined with the detection speed as a criterion for rating the models' goodness. The detection results of the three network models in pantograph faults are shown in Table 3, where the detection time is the average time of detection of all test samples in dataset 1.

From the detection results in Table 3, it can be seen that the faster R-CNN model based on DenseNet121 achieves an A*P* value of more than 92% for all types of pantograph states with only the original data set, which is more than 5% higher than VGG16 and about 1% higher than ResNet101, and in the detection of pantograph disconnection and bending faults, the DenseNet121 network is 2% higher than the ResNet101 network because DenseNet is able to extract deeper pantograph image features and has good overfitting resistance even in the case of small pantograph fault sample size. The detection speed is also faster than that of the ResNet101 network because the DenseNet network uses directly connected pantograph image features from different network layers in parallel, and each layer needs to learn fewer parameters; so, the detection speed of the DenseNet network is faster when the network layers are comparable.

## 5. Conclusion

By using the DenseNet network as a feature extraction network for the faster R-CNN model, which can extract deep-level image features and accomplish feature reuse, deep-level pantograph image features may be exploited, and the subway fault detection effect improved. The detection model is evaluated using pantograph images under various conditions such as multiple pantographs, in-tunnel and at night, and compared with the original model and the detection results based on the ResNet network model. The simulation results show that the method presented in this paper is more effective in pantograph fault detection, with a mean average accuracy of more than 4% higher than the original detection model, and a mean average accuracy of more than 98% after adding expanded samples, effectively addressing the problem of low detection accuracy in the case of fewer pantograph fault samples. In this paper, only the pantograph positioning and the detection of two obvious faults of broken wire and bending are realized, and further research on the detection of other pantograph faults will be conducted on this basis in the next step.

## Figures and Tables

**Figure 1:** Subway fault diagnosis system.

**Figure 2:** Subway fault handling process.

**Figure 3:** Pantograph schematic.

**Figure 4:** Model architecture.

**Figure 5:** Schematic diagram of densely connected network.

**Figure 6:** Schematic diagram of loss reduction during training.

**Figure 7:** Training process performance improvement schematic.

**Table 1:** Data information.

Sample	Datasets	zcdx	xbdx	dkdx
Dataset 1	Total number	856	206	223
	Training set	599	144	156
	Test set	257	62	67

Dataset 2	Total number	5992	1442	1561
	Training set	4194	1099	1093
	Test set	1798	433	468

**Table 2:** Classification information.

Real situation	Predicted results	
	Positive example	Counterexamples
Positive example	TP (true example)	FN (false counter example)
Counter example	FP (false positive example)	TN (true counterexample)

**Table 3:** Performance comparison.

Model	xbdx	dkdx	zcdx	Time	mAP
Faster + VGG16	91.30	86.30	88.40	0.23	88.67
Faster + ResNet101	95.30	90.50	94.30	0.33	93.37
Faster + DenseNet121	96. 10	92.90	96.30	0.20	95.10

## Data Availability

The datasets used during the current study are available from the corresponding author on reasonable request.
